# Optimization of Data Acquisition Link of University Students' Physical Health Testing System

**DOI:** 10.1155/2022/5343009

**Published:** 2022-01-25

**Authors:** Xiaohui Zhai, Yuanle Li, Chunli Zhong, Cheng Zhong, Yunke Luo

**Affiliations:** ^1^Physical Education Institute, Hunan University, Changsha, China; ^2^Physical Education College of Chongqing University, Chongqing, China

## Abstract

University students' physical health test is an important part of university physical education. The data obtained by the physical health test play an extremely important role in the field of students' physical health research. This paper clarifies the current situation of data collection of the physical health test for college students by sorting out the development status and trend of the physical health test system in China. To further ensure the accuracy and validity of the physical health test data, this article puts forward the corresponding optimization measures for the data collection link of the existing physical health testing system given the problems existing in the implementation of university students' physical health tests. Optimization measures are as follows: (1) add a test data collection type for test video collection; (2) optimize the authentication process to increase face recognition; and (3) enhance posttest test data management by stamping time.

## 1. Introduction

The physical health of teenagers has always been the focus of countries. Countries have issued relevant policies and systems to escort the development of teenagers' physical and mental health. The physical health test is an important means to examine the physical health of students, and the test results are also an important indicator to judge the physical health of teenagers [1]. The data can provide the guiding basis for the establishment of a follow-up system and the determination of work direction. China has successively formulated many systems to promote the development of physical health testing. And these policies and systems enable students to have a clearer evaluation standard for their physical health such as <The National Students' Physical Health Standard> and <The Measures For The Monitoring And Evaluation Of Students' Physical Health>.

## 2. Physical Health Test Data and Physical Health Testing System

There are some problems in Chinese students' physical health test data, such as waste of data resources and single application path [2]. Most of the physical health test data in colleges and universities are only submitted to the superior departments or issued reports and feedback, but not further application. Physical health test data play an extremely important role in the field of students' physical health. Real and effective physical health test data can ensure the smooth development of physical health research and accurate judgment, the application of physical test results, and the effectiveness of research results. The accuracy and authenticity of physical health test data are closely related to whether the data collection is scientific and rigorous [3] and whether the data have been modified after data collection [4]. The physical health testing system (or physical health test management system) is an intelligent test system serving for physical health testing. The existing physical health testing system is mainly for students of all grades. The physical health testing system generally consists of data acquisition and transmission module, a communication and transmission module, a data calculation and service module, and an application and management module. The data acquisition equipment of some physical health testing systems is also different according to the different service objects. The physical health testing system relies on a variety of intelligent devices and intelligent terminals for data collection. The data collected by the physical health testing system are directly transmitted to the server through a wireless network. Then, proceed to the next step of error data screening, correction, calculation, analysis of results, and storage. Finally, the system user carries out test management, data management, and other operations through the system platform of the terminal or app software. Therefore, aiming at the problems found in the process of the university students' physical health test, we start with the data acquisition link of the university physical health testing system. The accuracy and authenticity of physical health data is improved by the optimization of the university students' physical health testing system.

## 3. Development Status of Physical Health Testing System at Home and Abroad

China's student physical health testing system was developed late. FITNESSGRAM, a computer information management system based on fitness test reports, was developed in 1977 in the United States. Its development concept is to realize the whole process of integrating physical health tests into physical education. Therefore, the system attaches great importance to the students' physical health service and feedback on the result after the test [5]. China launched the student physical health standard intelligent service system in 2003, which is mainly used for the reporting, statistics, and calculation of physical health test data [6]. The development concept of the system is the information management of data, so the system lacks the follow-up student physical health service and feedback function [7].

However, the China's physical health testing system has developed rapidly in recent years. Many scholars pay attention to the cross integration of disciplines and apply advanced technologies in various fields to the physical health testing management system to promote the intelligent development of the system, such as the physical health testing management system designed based on a variety of wireless transmission modules, computer vision technology, and mobile Internet technology [8–10]. A variety of intelligent testers are designed based on infrared detection systems for physical health test data acquisition [11, 12] and physical health test data analysis systems or software based on different algorithms [13, 14]. The integration of artificial intelligence, computer software engineering, big data, medicine, and sports in the new engineering makes the physical health testing system develop rapidly and the function of the system more comprehensive.

At present, there are mainly two types of physical health testing systems in the Chinese market. And there are great differences in data acquisition modules between the two types of systems.

A full set of intelligent testing equipment is used for intelligent data collection without manual input. For example, the smart sports management platform [14] was designed by Best Technology Co., Ltd, which collects data through intelligent test equipment. The other is to collect data through the handset, which needs manual tests and input. For example, Henan Ding Huixin Network Technology Co., Ltd. designed a physical health testing system that relies on physical testing handheld devices for data collection.

At present, the research focus of the physical health testing system in China mainly includes the collection and management of sports health testing data, and the follow-up health service and feedback are also being further studied. The tentative application of these advanced and innovative research methods has greatly improved the efficiency and safety of students' physical health testing in China.

## 4. Problems Existing in the Data Acquisition Module of the Physical Health Test of College Students

There are many deficiencies in the process of physical health tests for university students, which affect the accuracy, authenticity, and diversity of physical health test data. The application of the university students' physical health testing system can make the data collection of physical health testing more accurate and convenient. However, the system still fails to effectively prevent and solve the problems in the physical health test of university students.

### 4.1. Physical Health Testing Data Collection Type Is Single

Data are not just numbers; they also contain text, images, sounds, and so on. However, the data collection of most of the students' physical health testing systems in the market is limited to the student's test scores, that is, digital collection [15, 16]. Only collecting numbers in the physical health test cannot meet the needs of the current student's physical health promotion work. Numbers can reflect the changes in students' grades, but we cannot judge whether students' body posture is normal or whether their motor skills are correct according to numbers. At present, the follow-up service of students' physical health is no longer just a simple treatment and feedback of test scores, but more important is to issue personalized exercise prescriptions according to students' physical conditions and sports characteristics. In this way to promote students to participate in the exercise, enhance students' physique, especially in the field of science and technology to help develop teenagers' physical health, a variety of sports apps, smart wearable devices, sports prescription systems, sports clothes, and others emerging in an endless stream. The proposal and development of an online sports prescription expert system [7] put forward higher requirements for the diversification of data collection types. The physical characteristics and technical movements of the subjects had an impact on the issuance of exercise prescriptions. However, there is a lack of diversity in the data collection types of physical health tests for university students. Most of them are limited to the collection and uploading of test results.

### 4.2. Loose Authentication Procedures during Physical Health Testing

Now the physical health test is linked with academic credits, evaluation, and graduation qualification [17], and students' attitude towards the physical health test has changed. Most of the students can correctly understand the physical health test and improve their physical fitness by actively participating in physical exercise to pass the test or improve the test results. However, there are still some students with cognitive errors, neglect exercise, and take shortcuts to complete the physical health test such as the behaviors of the substituting test.

The existing data acquisition module of the university students' physical health testing system are generally equipped with student card verification or test card verification device. The test worker can read the identity information before the test. However, the lax management of the testing process and the negligence of identity verification [18] have led to loopholes for students to follow. For example, proxy exam takers often succeed because the staff does not strictly verify whether the holder and certificate are consistent during the test. Proxy exam takers only need to hold their student id cards to take the test.

### 4.3. The Test Data Is Distorted

In 2004, the Ministry of Education of China began to build a large-scale national information system of students' physical health test data to cooperate with the national students' physical health standards. And schools at all levels across the country are required to report their students' physical health test results to the Ministry of Education. So some local education authorities have created incentives to promote physical fitness testing. For example, if the average score of the students' physical health test decreases for two consecutive years or the myopia rate increases for two consecutive years, the evaluation of their performance of educational responsibilities shall be reduced by one grade [19]. To avoid degradation and be criticized, some schools sorted out and calculated the physical health test data of the current year in advance for “optimization and adjustment” because their physical health scores were not ideal [20]. These practices lead to great differences between self-test data and later spot check and review data, and the authenticity of self-test reported data is questionable [21].

Although the existing physical health testing system of university students reduces manual operation as far as possible in the process of data collection, transmission, and uploading to the national database, it does not take effective measures to monitor the data. System operators can still modify the original data at will without any modification record. As a result, the authenticity of the data in the national student physical health standard database is doubtful, which cannot meet the purpose and target of the test.

## 5. Optimization Countermeasures of Data Acquisition in the Physical Health Testing System

### 5.1. Enriching Test Data Collection Types: Test Video Collection

The existing moving video image acquisition methods are divided into plane acquisition, three-dimensional acquisition, high-speed acquisition, multimachine acquisition, and infrared acquisition, and so on. Among them, the plane acquisition is the main way of motion video image acquisition. The plane image acquisition is divided into plane fixed-point focus acquisition, plane fixed-point zoom acquisition, plane fixed-point focus scanning acquisition, plane fixed-point focus moving acquisition, and plane zoom moving acquisition. [22] There are 8 physical fitness tests for university students in China, including 50 meter run, sitting forward bending, standing long jump, height, weight, vital capacity, pull-up (sit-ups for girls), and 1000 meter run (800 meter run for girls).

#### 5.1.1. Each Project Tested the Video Capture Method

In sit and reach, standing long jump, vital capacity, sit-ups, and chinning, the movement range of the subject is small. So the plane fixed-point focus acquisition method is used for test video acquisition. The moving video image is carried out through the fixed-position video recording device, and the real-time control of the device and the remote transmission of the moving video image are realized in combination with the wireless multimedia sensor network technology, controller, and terminal equipment. The plane fixed-point and fixed focus acquisition method requires that the camera shooting distance shall not be less than 25 m and the field width shall not be less than 8 m. [22] Therefore, when these projects are tested, only one stand is needed to realize moving video image acquisition.

The subjects moved a wide range during the 50-meter race, the 800-meter race, and the 1,000-meter race. Therefore, in track and field competition, the planar fixed focus mobile acquisition method is generally adopted. However, this kind of collection method needs to use slide track technology and install slide track inside or outside the runway. Then, install a video acquisition device on the slide track for video acquisition. However, this method has a high cost, so it is suggested to adopt a multipoint plane fixed focus acquisition method to acquire moving video images under the comprehensive consideration of the testing cost and other factors. Among them, the fixed-point shooting positions of 800 m and 1000 m are the starting point, 200 m curve, and the end point. The three points collect the subjects' starting video, curve running video, and sprint running video, respectively. The 50 m running distance is short and the movement path is a straight line, so it is selected to shoot at the starting point and the end point. Students' starting action videos are collected at the starting point, and students' enroute running action videos are collected at the end point. This method can obtain the motion characteristics of the subjects in different stages, and the video can be used to verify whether the testers participate in the whole test.

The acquisition of test videos can meet the needs of the following three aspects: first, the demand for supporting materials during random inspection and review of the physical health test. By watching and checking the test video, we can verify whether the students' test results are true and whether the school test process is qualified. The second is the follow-up management service demand of the physical health test. Rich and diverse physical health test data can support the development of sports guidance, health research, and judgment. Third, science and technology help develop the needs of teenagers' physical health. Video data can provide a data basis for the research and development of intelligent wearable devices, sports apps, sportswear, etc., as shown in Figure 1.

### 5.2. Optimizing Authentication Link: Face Recognition Technology

Biometric identification has the highest security and reliability among the existing identification technologies. Common biological features are divided into physiological features—face, DNA, fingerprint, iris, etc.; and behavioral features—gait, voice, signature, keystroke habit, etc. Among them, face recognition technology is a noncontact recognition technology. Compared with fingerprint verification, iris authentication, and other recognition technologies, it has the advantages of being fast, simple, high reliability, difficult to counterfeit, low cost, and noncontact. In particular, the active resolution of face recognition technology ensures that others cannot be recognized by the system when using nondynamic picture puppets and wax figures. Therefore, adding facial recognition to the test equipment can not only ensure that the identity of the subject is correct but also avoid the subject using pictures and other deceptive.

Face recognition technology collects face pictures or videos for identification and authentication. Identification is to check the collected image and the image in the face database to confirm the identity information. Identity authentication is to check the image with the photo in the ID card to determine whether it is the same person.

This article adopts identity authentication, that is, to judge whether two face images belong to the same identity. During the test, the subject swipes the student card to obtain his basic information and then verifies whether the student is the subject through face recognition.

#### 5.2.1. Selection of Face Recognition Algorithm

Face recognition technology integrates artificial intelligence, machine learning, video image processing, and other professional technologies and is the latest achievement and application of biometric technology. Face recognition is to use a camera to collect the image or video of the face, and automatically detect and track the face in the image, and then compare the detected face image, detection, and a series of related operations. In the physical fitness test, multiple test items are performed outdoors. However, the outdoor light is changeable and the environment is complex. Compared with document photography, the images obtained by face recognition camera in the test are very different in light, human behavior, posture, expression, and other aspects.

SeetaFace is characterized by complete code, convenient transplantation, and optimization, which can meet the needs of lightweight face recognition, and it uses the five-point location method in the feature point location module, which greatly reduces the amount of calculation. Therefore, the SeetaFace face recognition engine is selected as the basic algorithm for face recognition. The automatic face recognition system needs three basic modules: face detection module, face feature point positioning module, and face feature extraction and comparison module. However, the small number of registration points will lead to the problem of inaccurate positioning in the case of low resolution or large facial offset angle. But, in physical health tests, subjects are usually fixed in front of data acquisition equipment for identity authentication, so the large facial offset angle can be controlled. At the same time, the resolution of the assembled camera is high enough to solve the resolution problem. Most importantly, the reduction in computation demands less on the processor and therefore costs less. Therefore, this method is suitable for face recognition of the data acquisition module of the physical health testing system.

#### 5.2.2. Authentication Process of the Physical Health Testing System Data Acquisition Module

Before the test of a project, the subject first reads the student card information at the information reading place of the test equipment of the project (including the student's ID photo). The face recognition camera will get the image, and the student card information of the personal ID photo will be compared to confirm whether it is the same person. Finally, according to the different certification results to decide whether continue the test, the specific process is shown in Figure 2.

### 5.3. Strengthening Test Data Management: Data Tamper-Proof Technology

At present, the data collection of the physical health testing system has been automated. And it is impossible to modify a large number of data in this link. However, it is still possible to modify the data manually in the data upload and data reporting stage after data collection. Therefore, the tamper-proof of physical health data needs to start from the source and take corresponding measures in the stage of data collection and uploading to ensure the primitiveness of data. There are many tamper-proof technologies for electronic data: document solidification technology, digital signature technology, trusted timestamp technology, blockchain technology, and so on.

#### 5.3.1. Choice of Data Tamper-Proof Technology

The physical health test of students covers a wide range, and the amount of data obtained is huge. In addition, the authenticity and validity of test data plays an extremely important role in promoting students' physical health in China, so it is necessary to choose an economical and effective way to ensure the authenticity and originality of test data. The technology has strong operability and can effectively play a role in data security protection.

Timestamp technology is a technology that uses the hash algorithm and asymmetric encryption algorithm to verify the originality and authenticity of data with the help of the time proof of the third-party timestamp mechanism. It has strong operability and can effectively protect the data. Timestamp technology has been applied in many fields, such as archive data management, traffic law enforcement, accident handling, food traceability, criminal investigation of public security organs, and so on. The generation of the timestamp is realized by three parties, namely, the users, national timing center, and time stamp organizations, so its reliability is strongly guaranteed. And because it can track the whole process of data, it can ensure the validity and reliability of data.

Using this technology in the physical health testing system can control the source of testing data and the whole process of testing data development. Users can track the query, modify, delete, and use records of test data to realize the whole process monitoring of test data. Therefore, data tampering can be prevented and the reliability of test data is guaranteed.

#### 5.3.2. Timestamp Timing Selection

It is necessary to select the appropriate time for stamping the time stamp, as early or late stamping can adversely affect test data. Students' physical health test items are diverse, the number of test people is large, and the test data generated is huge. If each project's test data or each person's test data are time-stamped, more data will be generated and too much memory will be occupied and resources will be wasted. Therefore, after the physical health test was completed on the day, the supervisors of the third-party supervision organization stamped the physical health test data. General physical fitness testing will continue for several days. The timestamp at the end of each test can ensure the reliability of data and avoid the data burden caused by too many time stamps, as shown in Figure 3.

## 6. Deficiencies of This Research

This article puts forward some problems existing in the physical health testing system of university students and puts forward optimization countermeasures for these problems, but there are still deficiencies in some areas, which are given as follows:

1. The timestamp technology selected in this article has high requirements on the third-party supervisory organization, because the time stamp needs to be strictly implemented and grasped by the third-party supervision organizations. But at present, the independence of the third-party supervisory organization in our country is not enough and the laws and regulations are absent [23]. It needs to be constantly strengthened.
2. The data storage problem is unresolved. Video data take up more memory than pure digital data, so reducing memory consumption is also extremely important in system development. In this respect, relevant professionals are needed to further optimize.

## 7. Conclusion

The intelligent student's physical health testing system is the product of the progress of times and also the development direction of the student physical health testing system in the future. Providing scientific and comprehensive health guidance for students, promoting the development of lifelong physical education, and finally realizing the wisdom of physical health management are the ultimate goals of the physical health testing system. Accurate and true physical health test data can not only reflect the real physical condition of current Chinese college students and provide a solid data basis for the formulation of national policy documents, but also promote the development of follow-up service modules of the physical health test system and guide students to do physical exercise more accurately and scientifically. Therefore, this study starts by optimizing the data acquisition module of the physical health testing system to achieve a more accurate and comprehensive acquisition of students' physical health data, provide perfect information support for the follow-up service of physical health tests, and promote the healthy development of students' physical health.

## Figures and Tables

**Figure 1:** Location diagram of video recording equipment.

**Figure 2:** Face recognition workflow.

**Figure 3:** Timestamp application flow chart.

## Data Availability

The datasets used and/or analyzed during the current study are available from the corresponding author on reasonable request.
